# Effect of Perioperative Comprehensive Nursing Intervention on Transcatheter Arterial Chemoembolization in Patients with Primary Hepatic Carcinoma

This article has been retracted.

**DOI:** 10.1155/2022/9000331

**Published:** 2022-06-29

**Authors:** Min Hu, Ziyan Fan, Yu Han

**Affiliations:** ^1^Department of Surgical Special Needs Ward, Lu'an Hospital of Anhui Medical University, Lu'an, China; ^2^Department of Health Management Center, Lu'an Hospital of Anhui Medical University, Lu'an, China

## Abstract

**Objective:**

To study and analyze the effect of perioperative comprehensive nursing intervention on transcatheter arterial chemoembolization (TACE) in patients with primary hepatic carcinoma (PHC).

**Methods:**

One hundred and ten patients with PHC diagnosed in our hospital from May 2019 to January 2022 were randomly selected and divided into a control group (*n* = 55) and an observation group (*n* = 55) by random number sorting according to odd and even numbers. Patients in the control group received conventional nursing interventions and those in the observation group received comprehensive nursing interventions. The two groups were compared in terms of surgical status, quality of life (QoL), and nursing satisfaction.

**Results:**

The operation time, postoperative bed rest time, and hospital stay in the observation group were significantly (*P* < 0.05) shorter than those in the control group; the observation group had significantly (*P* < 0.05) higher scores of quality of life, including somatic function, emotional function, role function, social function, and cognitive function than the control group; chemotherapy adverse reactions including fever, abdominal pain, urinary retention, and gastrointestinal reactions in the observation group were significantly less than those in the control group (*P* < 0.05); the total incidence of complications in the observation group was significantly (*P* < 0.05) lower than that in the control group. The total satisfaction with nursing care in the observation group was significantly (*P* < 0.05) higher than that in the control group.

**Conclusion:**

The perioperative application of comprehensive nursing intervention in TACE for patients with PHC aids in the smooth operation, improves patients' QoL, lowers the risk of chemotherapy reactions and complications, and enhances patient satisfaction and nursing quality. These advantages justify a wider perioperative application of comprehensive nursing intervention in TACE clinical practice.

## 1. Introduction

Primary hepatic carcinoma (PHC) refers to a malignant tumor occurring in hepatocytes or intrahepatic cholangiocytes [1]. Recent years have witnessed the rising incidence of PHC across the globe. Hepatic carcinoma has been more common in men over 40 years old in China, according to relevant epidemiological statistics, with a male-to-female incidence ratio of roughly 2.7 : 1 [2]. Its histopathological types include hepatocellular carcinoma, cholangiocarcinoma, mixed cellular carcinoma, and other special types. Among them, hepatocellular carcinoma accounts for more than 80% and cholangiocarcinoma represents about 5%–10% [3]. Mixed cellular carcinoma is uncommon and rarer even are such particular types as fibrolamellar carcinoma and clear cell carcinoma [4]. Most of the clinical symptoms include hepatomegaly, liver pain, systemic and gastrointestinal symptoms (such as fatigue, emaciation, inappetence, and abdominal edema), and metastatic liver cancer symptoms. However, as the disease is in its early stages, patients exhibit typical clinical signs and symptoms usually in the middle to late stages, when they are asymptomatic and have an insidious onset [5]. The prognosis of hepatocellular carcinoma is largely dependent on early diagnosis and treatment. The 5-year survival rate is 30–50% after resection for hepatocellular carcinoma and 50–60% after resection for small hepatocellular carcinoma [6, 7]. In summary, PHC is a common malignant tumor in China and causes a lot of suffering to people.

PHC treatment is defined by the convergence of several approaches and disciplines in clinical practice, with a focus on interdisciplinary comprehensive care and individualized treatment. The main treatment approaches include hepatectomy, liver transplantation, local ablation, transcatheter arterial chemoembolization (TACE), radiotherapy, and systemic drug therapy. TACE is an interventional therapy that primarily involves femoral artery intubation and sending anticancer drugs or embolic agents into the hepatic artery [8, 9]. This technique is only applicable to patients with hepatic carcinoma and is currently the top choice for nonsurgical treatment of hepatic carcinoma [10, 11]. It can not only kill tumor cells directly but also cut off the tumor's blood supply, causing it to “starve to death” without nutrition. Using the Seldinger puncture and cannulation technique, the hepatic artery is routinely punctured through the right femoral artery, and celiac arteriography is routinely performed. If it is found that the tumor vascular tumor staining is incomplete, continue to search for variant blood supply arteries [12–14].

Previous research findings reveal that TACE can not only lengthen patients' lives and control disease progression but also pave the way for secondary surgical treatment [15]. However, many clinical practice results suggest that TACE can cause a series of chemotherapeutic responses and complications, as well as varying degrees of liver reserve function impairment [16]. Therefore, active and effective nursing intervention techniques for patients in the perioperative period are essential for the prevention and management of chemotherapeutic reactions and complications as well as the protection of liver function [17, 18]. The aim of this study was to investigate and evaluate the impact of comprehensive perioperative nursing interventions on TACE in patients with PHC, providing a reference value and theoretical basis for future clinical practice.

## 2. Materials and Methods

### 2.1. Subjects

A total of 110 patients who were diagnosed with PHC and received TACE in our hospital from May 2019 to January 2022 were randomly selected, including 81 males and 29 females, aged between 43 and 75 years, with a mean age of 60.34 ± 9.84 years. All patients were allocated to the control group (*n* = 55) and the observation group (*n* = 55) according to odd and even numbers through random number sequencing. Patients in the control group were treated with routine nursing intervention, while patients in the observation group received comprehensive nursing intervention. Their families and themselves were informed of the study and signed the informed consent form voluntarily. The experiment has been approved by the ethics committee of our hospital (Approval ID: 20190420).

### 2.2. Inclusion and Exclusion Criteria

  Inclusion criteria: (1) patients who met the diagnostic criteria for PHC; (2) patients who received TACE treatment; and (3) patients with no distant metastasis found in clinical examinations.
  Exclusion criteria: (2) patients with severe heart, lung, liver, and renal insufficiency; (2) patients with mental illness or unconsciousness; and (3) patients with complications such as severe jaundice or abnormal coagulation function.

## 3. Methods

Patients in both groups were treated with TACE after being diagnosed and admitted to the hospital [19]. They received the following treatment: preoperative preparations were routinely performed. All patients were placed in the supine position. Local anesthesia was performed before the operation, and the puncture point was disinfected. The Seldinger maneuver was used to puncture the femoral artery, and the 5F-RH catheter or Yashiro catheter was inserted into the celiac artery or common hepatic artery for DSA. Angiography was performed to determine the location, size, number, and supplying arteries of the tumor and then perfusion with chemotherapy drugs, often using epirubicin, lobaplatin, or oxaliplatin, 5-fluorouracil (5-Fu), etc., 2–3. According to the patient's tumor burden, body surface area, physical fitness status, previous drug use, and whether it is used in combination, the compatibility and dosage should be selected, and the infusion time of chemotherapy drugs should not be less than 20 minutes. The ultraliquefied lipiodol and chemotherapeutic drugs were fully mixed into an emulsion, and then, chemoembolization was performed under fluoroscopy. After completion, routine angiography was performed to monitor the state of embolization. After surgery, normal pressure was applied to the puncture site with a bandage for 12 hours. 

Patients in the control group received routine nursing intervention, including observation of illness, improvement of preoperative examination, medication guidance, routine dressing change at the puncture site, bandaging, and prevention of infection.

Patients in the observation group were treated with comprehensive nursing intervention. Specific treatment included the following:

1. Before the operation, patients were informed of relevant information to allow them to fully and correctly understand the etiology, clinical manifestations, treatment methods, and prognosis of cancer. Any discomfort and complications that may occur after operation were explained in detail. According to the individual situation of patients, appropriate psychological care and health guidance were formulated, and a relationship of mutual trust with patients was established for patient encouragement and compliance as well as the elimination of negative emotions such as anxiety, fear, depression, and sadness that often appear in the treatment process. Preoperative guidance and preparation of surgical instruments and drugs were conducted, followed by a detailed physical examination and allergy tests. Patients were reminded to fast 4 hours before the operation.
2. Intraoperative: patients cooperated with physicians to complete the operation, with the indexes of patients normally checked and the internal conditions of patients monitored. Patients were informed of the chemotherapy process promptly. Physicians could remind patients to be mentally prepared before injection chemotherapy, which may cause obvious discomfort. They could also tell patients that the operation was successful and praise the patient's compliance when it was approaching the end of the operation. Various conditions should be handled reasonably appropriately: pain care, attention to control, respiratory control, and position adjustment to relieve the patient's pain. Patients in severe pain may be given analgesics to relieve severe pain with the consent of the physician's diagnosis. Nursing for complications and adverse reactions was performed with prevention in advance by ventilating and maintaining a warm temperature in the ward, frequently changing sheets and clothes, closely monitoring the condition, and timely handling the side effects and complications of chemotherapy to different degrees. Diet nursing was followed according to the individual physiological and dietary characteristics of patients, with reasonable and healthy daily diet plans formulated, and the diet plans focused on light foods with high calorie, high cellulose, and high protein, boosting the patients' body resistance and immunity. Daily life nursing intervention was conducted through formulating activity plans according to the actual situation of patients after operation, such as encouraging patients to get out of bed for postoperative recovery, paying attention to sleep quality, guiding patients to rest more, drinking water properly, sleeping well, carefully following the doctor's instructions on medication, and regularly checking liver function and blood circulation [20].

### 3.1. Evaluation Criteria

1. Detailed recording and comparison of the two groups, including the duration of surgery, postoperative bed rest, and length of hospital stay.
2. QoL rating scale (SF-36) was used to evaluate patients' quality of life, which was divided into five dimensions: somatic function, emotional function, role function, social function, and cognitive function. The total score of each dimension was 100 points. The higher the score after evaluation, the better the patient's quality of life.
3. Chemotherapy adverse reactions, including fever, abdominal pain, urinary retention, and gastrointestinal reactions, were recorded in detail and compared between the two groups.
4. We also recorded and compared the complications of the two groups, including renal failure, tumor rupture, hemorrhage of the digestive tract, and puncture point bleeding. The total incidence of complications was calculated and compared between the two groups. Complication rate = number of people with complications/total number × 100%
5. Using the Questionnaire of Nursing Satisfaction created by our hospital (for the evaluation of medical personnel from the perspectives of attitude, efficiency, and disease explanation, among others), we set four options of satisfaction (very satisfied, satisfied, not very satisfied, and dissatisfied) to understand the satisfaction of the two groups of patients and determine which one of the two groups of treatment methods was more effective through the results.

### 3.2. Data Analysis

The GraphPad Prism 8 software was used to process images, and data processing was conducted with the SPSS 22.0 software. Chi-square tests and *t*-tests were performed for enumeration data (*n* (%)) and measurement data ($\bar{x}$ ± *s*), respectively. The difference was statistically significant if *P* < 0.05.

## 4. Results

### 4.1. General Data

In the control group, there were 55 cases, including 41 males and 14 females, aged 43–75 years, with a mean age of 61.25 ± 9.24 years. The course of the disease was 0.5–7.1 years, with a mean course of disease of 3.53 ± 1.78 years. The diameter of the carcinoma was 5–13 cm, with a mean diameter of 7.82 ± 1.71 cm. There were 55 cases in the observation group, including 40 males and 15 females, aged 43–75 years, with a mean age of 59.42 ± 9.72 years. The course of the disease ranged from 0.8 to 7.5 years, with a mean course of disease of 3.68 ± 1.74 years. The carcinoma diameter ranged from 5 cm to 13 cm, with a mean diameter of 7.68 ± 1.84 cm. There was no significant (*P* > 0.05) difference in general data between the two groups, but the two groups were comparable. See Table 1 for details.

### 4.2. Operation Situation

The operation time, postoperative bed rest time, and hospital stay in the observation group (66.78 ± 13.25, 39.48 ± 5.65, 9.08 ± 1.23) were significantly (*P* < 0.05) shorter than those in the control group (75.69 ± 18.65, 47.38 ± 5.98, 11.23 ± 2.17). See Table 2 for details.

### 4.3. QoL

The observation group had significantly (*P* < 0.05) higher scores of QoL, including somatic function, emotional function, role function, social function, and cognitive function (84.51 ± 11.25, 86.68 ± 10.17, 84.45 ± 11.52, 83.45 ± 11.51, 84.64 ± 10.54) than the control group (69.17 ± 15.56, 68.91 ± 12.56, 67.45 ± 13.34, 69.08 ± 15.56, 66.98 ± 15.68). See Table 3 for details:

### 4.4. Chemotherapy Adverse Reactions

Chemotherapy adverse reactions including fever, abdominal pain, urinary retention, and gastrointestinal reactions (12 (21.82%), 15 (27.27%), 8 (14.55%), 10 (18.18%)) in the observation group were significantly (*P* < 0.05) less than those in the control group (39 (70.91%), 32 (58.18%), 28 (50.91%), 31 (56.36%)). See Table 4 for details.

### 4.5. Complications

There were 0 (0.00%) case of renal failure, 0 (0.00%) case of tumor rupture, 1 (1.82%) case of hemorrhage of the digestive tract, and 2 (3.64%) cases of puncture point bleeding in the observation group, while 5 (9.09%) cases of renal failure, 0 (0.00%) case of tumor rupture, 7 (12.73%) cases of hemorrhage of the digestive tract, and 6 (10.91%) cases of puncture point bleeding in the control group. The total incidence of complications in the observation group (5.45%) was significantly (*P* < 0.05) lower than that in the control group (32.73%). See Table 5 for details.

### 4.6. Satisfaction

The results of questionnaire survey showed that 15 (27.27%) patients in the control group were very satisfied, 25 (45.45%) were satisfied, 11 (20.00%) were not very satisfied, and 4 (7.27%) were dissatisfied. In the observation group, 26 (47.27%) patients were very satisfied, 28 (50.91%) were satisfied, 1 (1.82%) was not very satisfied, and 0 (0.00%) was dissatisfied. The total satisfaction with nursing care in the observation group (98.18%) was significantly (*P* < 0.05) higher than that in the control group (72.73%). See Figure 1 for details.

## 5. Discussion

Primary liver cancer has become the fourth most common malignancy and the second leading cause of death in China, posing a serious threat to human safety and health [21]. The etiology of primary liver cancer is not fully understood and may be the result of a synergistic effect of multiple factors. Based on epidemiological investigations, it is mostly believed to be related to the following susceptibility factors. About 70% of primary liver cancers occur on the basis of cirrhosis, and most of them are nodular cirrhosis that develops from chronic hepatitis B and C [22]. The risk of liver cancer is greater when HBV or HCV infection coexists with alcoholic or nonalcoholic fatty liver disease [23]. Hepatic encephalopathy is a terminal complication of primary liver cancer and accounts for one third of the causes of death. Another is gastrointestinal bleeding, which accounts for approximately 15% of the causes of death from liver cancer [24]. Combined cirrhosis or portal vein or hepatic vein carcinoma embolism can lead to ruptured oesophagogastric fundic varices and bleeding [25]. Secondary infections are due to long-term consumption of cancer, especially in the case of reduced white blood cells after radiotherapy and chemotherapy, weakened resistance, coupled with factors such as prolonged bed rest, which can easily complicate various infections, such as pneumonia, intestinal infections, and fungal infections [26].

TACE is a combination of medical imaging and clinical treatment that has become one of the most important treatments for the treatment of PHC, as it can help reduce tumor volume and allow for a second operation. Although liver resection or transplantation provides better results than other therapies in the local control of HCC, survival rates are unsatisfactory, particularly for large tumors, and it remains controversial whether HCC angiogenesis is enhanced after TACE even in patients undergoing radical resection [27]. It is frequently utilized in arterial infusion chemotherapy with chemotherapy drugs that are generally given all at once at a high concentration and large dose. The drugs selected in this study have been verified and confirmed in clinical practice that they can affect microtubules of cells and promote aggregation, thus preventing microscopic aggregation and rearrangement, inhibiting mitosis, interfering with tumor cell dynamics, and effectively preventing tumor cell dissociation [28]. The perioperative period covers the entire period from the patient's admission to the surgical ward to the patient's postoperative recovery and discharge, i. e., the time before, during, and after surgery. At different stages of the perioperative period, the patient exhibits different signs. As the condition progresses, it creates a variety of problems. If patients are adequately prepared before and during the perioperative period, have a proper understanding of their psychological and physical condition, and take appropriate measures, they can be assured of better surgical treatment. Combined with reasonable and appropriate overall interventions during and after surgery, this will not only improve the overall treatment outcome but also effectively prevent various side effects and complications for patients, enabling them to complete their treatment and recover as soon as possible.

Previous studies have revealed that TACE for patients with PHC has noticeable adverse effects, such as digestive system reactions, that affect postoperative recovery and treatment effectiveness [29]. Based on the aforementioned, 110 patients with PHC diagnosed in our hospital were selected at random and divided into two groups for this study. Throughout the perioperative period of different groups of patients, routine nursing and comprehensive nursing interventions were carried out to ensure the smooth course of TACE and the realization of the intended results. The results showed significantly shorter operation time, postoperative bed rest time, and hospital stay in the observation group than those in the control group. Through an investigation of the reasons, comprehensive nursing intervention is considered to necessitate preoperative guidance to patients in a variety of ways, dispelling patients' uncertainties about diseases and treatment techniques, and assisting patients in fully and correctly understanding cancer. Measures such as improving the ward environment and keeping patients informed of the progress of the procedure can help to minimize the impact of numerous factors on the course and outcome of TACE in the perioperative period, thereby improving patient intraoperative indicators. The reduction in operative time suggests that comprehensive nursing interventions can improve the efficiency of medical staff and clinical turnaround rates. This is consistent with the findings of Zhao et al. The reduction in postoperative bed rest and hospital stay was mainly associated with the occurrence of adverse effects and complications of postoperative chemotherapy. In this study, it was observed that the observation group had significantly fewer adverse chemotherapy reactions and a significantly lower overall complication rate than the control group.

TACE has been shown to have positive efficacy. However, clinical controversy remains due to the necrosis of normal liver segments or lobe tissue in patients after occlusion of the liver donor vessels and the toxic side effects of chemotherapeutic drugs and embolic agents. The patient's postoperative recovery and overall treatment outcome are affected by a variety of adverse effects or complications. The application of comprehensive nursing intervention in the perioperative period requires postoperative nursing of complications and adverse reactions, which can be prevented in advance by ventilating and keeping warm in wards as well as changing sheets and clothes frequently. In the case of adverse reactions, medical staff will monitor the situation closely so that chemotherapy-related side effects and complications of varying degrees of severity can be managed promptly. This approach is effective in reducing the risk of chemotherapy reactions and complications for patients, as well as preventing patients from being bedridden, hospitalized for observation, or treated for adverse reactions and complications. The results also demonstrated that the observation group had significantly higher scores of QoL and total satisfaction with nursing care than the control group.

The physical pain, organ damage, and negative emotions associated with PHC may increase the risk or exacerbate the extent of adverse reactions. Also, due to the technical aspects of TACE and the physical condition of the patient, one or more adverse chemotherapy reactions and complications often occur after the procedure, leading to a variety of negative emotions and a significant deterioration in the patient's quality of life. However, comprehensive nursing interventions are required throughout the perioperative period, which means that care should be provided before, during, and after the procedure. Pain care alleviates the patient's suffering. Dietary care improves the patient's immune system. Daily life nursing intervention encourages patients to get out of bed for postoperative recovery, guides patients to rest more, drink enough water, and sleep well. Patients are instructed to carefully follow the doctor's advice on medications and regularly check liver function and blood circulation. It not only satisfies patients' needs for love and belonging, eliminates negative emotions, and increases patients' confidence and compliance in treatment, but it also improves their QoL, contributing to a considerable increase in patient satisfaction. This is consistent with the findings of Li et al., who found that perioperative comprehensive nursing could improve patients' psychosocial and self-care abilities, followed by a higher QoL [30].

## 6. Conclusion

To sum up, the perioperative application of comprehensive nursing intervention in TACE for patients with PHC aids in the smooth operation, improves patients' QoL, lowers the risk of chemotherapy resections and complications, and enhances patient satisfaction and nursing quality. These advantages justify a wider perioperative application of comprehensive nursing intervention in TACE clinical practice.

## Figures and Tables

**Figure 1:** Comparison of nursing satisfaction. ^*∗*^denotes that there is a statistically significant (*P* < 0.05) difference between the two groups.

**Table 1:** Comparison of general data ($\bar{x}$ ± *s*).

Group	Number of cases	Sex		Age (years)		Course of disease (years)		Tumor diameter (cm)	
		Male	Female	Range	Mean	Range	Mean	Range	Mean
Control group	55	41	14	43–75	61.25 ± 9.24	0.5–7.1	3.53 ± 1.78	5–13	7.82 ± 1.71
Observation group	55	40	15	43–75	59.42 ± 9.72	0.8–7.5	3.68 ± 1.74	5–13	7.68 ± 1.84
*t*	—	—	—	—	1.193	—	0.447	—	0.413
*P*	—	—	—	—	0.238	—	0.656	—	0.680

**Table 2:** Comparison of operation situation ($\bar{x}$ ± *s*).

Group	Number of cases	Operation time (min)	Postoperative bed rest time (h)	Hospital stay (d)
Control group	55	75.69 ± 18.65	47.38 ± 5.98	11.23 ± 2.17
Observation group	55	66.78 ± 13.25	39.48 ± 5.65	9.08 ± 1.23
*t*	—	2.888	7.121	6.392
*P*	—	0.005	<0.001	<0.001

**Table 3:** Comparison of QoL ($\bar{x}$ ± *s*).

Group	Number of cases	Somatic function	Emotional function	Role function	Social function	Cognitive function
Control group	55	69.17 ± 15.56	68.91 ± 12.56	67.45 ± 13.34	69.08 ± 15.56	66.98 ± 15.68
Observation group	55	84.51 ± 11.25	86.68 ± 10.17	84.45 ± 11.52	83.45 ± 11.51	84.64 ± 10.54
*t*	—	5.925	8.154	7.153	5.506	6.932
*P*	—	<0.001	<0.001	<0.001	<0.001	<0.001

**Table 4:** Comparison of chemotherapy adverse reactions (%).

Group	Number of cases	Fever	Abdominal pain	Urinary retention	Gastrointestinal reactions
Control group	55	39 (70.91)	32 (58.18)	28 (50.91)	31 (56.36)
Observation group	55	12 (21.82)	15 (27.27)	8 (14.55)	10 (18.18)
*t*	—	26.650	10.736	15.517	17.147
*P*	—	<0.001	0.001	<0.001	<0.001

**Table 5:** Comparison of complications (%).

Group	Number of cases	Renal failure	Tumor rupture	Hemorrhage of digestive tract	Puncture point bleeding	Total incidence
Control group	55	5 (9.09)	0 (0.00)	7 (12.73)	6 (10.91)	18 (32.73)
Observation group	55	0 (0.00)	0 (0.00)	1 (1.82)	2 (3.64)	3 (5.45)
*T*	—	13.242				
*P*	—	<0.001				

## Data Availability

No data were used to support this study.
